# A Holistic Performance Comparison for Lung Cancer Classification Using Swarm Intelligence Techniques

**DOI:** 10.1155/2021/6680424

**Published:** 2021-07-29

**Authors:** Sunil Kumar Prabhakar, Harikumar Rajaguru, Dong-Ok Won

**Affiliations:** ^1^Department of Artificial Intelligence, Korea University, Anam-dong Seongbuk-gu, Seoul 02841, Republic of Korea; ^2^Department of Electronics and Communication Engineering, Bannari Amman Institute of Technology, Sathyamangalam 638401, India; ^3^Department of Artificial Intelligence Convergence, Hallym University, Chuncheon, Gangwon 24252, Republic of Korea

## Abstract

In the field of bioinformatics, feature selection in classification of cancer is a primary area of research and utilized to select the most informative genes from thousands of genes in the microarray. Microarray data is generally noisy, is highly redundant, and has an extremely asymmetric dimensionality, as the majority of the genes present here are believed to be uninformative. The paper adopts a methodology of classification of high dimensional lung cancer microarray data utilizing feature selection and optimization techniques. The methodology is divided into two stages; firstly, the ranking of each gene is done based on the standard gene selection techniques like Information Gain, Relief–F test, Chi-square statistic, and *T*-statistic test. As a result, the gathering of top scored genes is assimilated, and a new feature subset is obtained. In the second stage, the new feature subset is further optimized by using swarm intelligence techniques like Grasshopper Optimization (GO), Moth Flame Optimization (MFO), Bacterial Foraging Optimization (BFO), Krill Herd Optimization (KHO), and Artificial Fish Swarm Optimization (AFSO), and finally, an optimized subset is utilized. The selected genes are used for classification, and the classifiers used here are Naïve Bayesian Classifier (NBC), Decision Trees (DT), Support Vector Machines (SVM), and *K*-Nearest Neighbour (KNN). The best results are shown when Relief-F test is computed with AFSO and classified with Decision Trees classifier for hundred genes, and the highest classification accuracy of 99.10% is obtained.

## 1. Introduction

The number of patients who are diagnosed with cancer is steadily increasing in a rapid manner [1]. With the help of biopsies, image processing techniques, and blood analysis, the diagnosis of cancer is done presently. When damaged cells are excessively accumulated in human body, it leads to cancer [2]. For every patient, the behavior of cancer differs, and by examining deeply into the origin of it, it can be well understood. The cancer originates in the cells and to every individual, the structure of the cell is quite unique. Therefore, to cure cancer permanently, there is not a single specific vaccine available [3]. Understanding the relation between the gene and its products is a contribution to the genetic approach to cancer diagnosis, so that the identification of biomarker genes for targeting drug therapies can be understood well [4]. With this approach, the effects of genes on some cell signaling pathways can be well understood [5]. The information about active levels of a gene is provided by the gene expression. For gene expression, one of the widely used measurement technique is microarray [6]. In the cancer diagnosis and cancer classification types, the gene expression values obtained by microarrays can be utilized. In many studies, the microarray datasets are employed for these purposes. For the selection of biomarker gene subsets, various feature selection algorithms are employed [7]. To this microarray dataset, statistic machine learning techniques are implemented with or without feature selection [8]. Biomarker genes are to classify cancer types, with a highest classification accuracy being identified by the biomarker genes.

In recent years, a new dimension to cancer research has been encompassed by the advent of microarray technology. For the classification, analysis, diagnosis, and treatment of cancer, a proficient method has been emerged by the microarray-based gene expression data [9]. Thousands of features termed as genes are found in the microarray gene expression dataset. Such data has records or instances from a few patients only and due to this limited availability of samples in comparison to larger number of genes, it is termed as curse of dimensionality problem [10]. Due to this, (a) the training time during the classification process is increased, and (b) there is a reduction in classification accuracy [11]. Therefore, the extraction of useful information from the dataset is hindered due to these challenging issues. So, the number of genes has to be reduced, and then, the highly informative genes should be selected, so that classification accuracy is increased, and it is a significant step in the microarray data analysis [12]. Feature selection/gene selection in the microarray data classification aim is to select a small subset of features from the original huge feature space [13]. By removing redundant and irrelevant features, feature selection can be done, so that the classification accuracy is increased, and the classification time is reduced. The feature selection technique proposed in the literature includes hybrid method, embedded technique, filter, and wrapper methods [14]. In this study, the primary aim is to classify and select the optimal gene subsets for lung cancer. Then, feature selection is implemented along with optimization techniques and finally classified.

Some of the prominent works in the lung cancer classification using microarray gene analysis are explained as follows. For the molecular classification of lung cancer, a cross study comparison of gene expression study was done by Parmigiani et al. [15]. Using the significance analysis of Microarray-Gene set reduction algorithm, the classification of non-small cell lung cancer was performed by Zhang et al. [16]. For multiclass classification of lung cancer, an adaptive multinomial regression with overlapping groups is performed by Li et al. [17]. The lung cancer prediction from microarray data by gene expression programming was done by Azzawi et al. [18]. A support vector machine-based classification method for lung cancer gene expression data base analysis was done by Guan et al. [19]. Some progresses in the techniques and integrated analysis related to the image processing techniques and the development of advanced devices for tissue engineering approach as a potential solution to treat lung diseases too have been discussed in the literature [20, 21].

As far as the microarray gene selection techniques using optimization and classification are concerned, self-organizing maps [22], ensemble classification techniques [23], Taguchi chaotic binary Particle Swarm Optimization (PSO) [24], adaptive wrapper approach combined with SVM [25], kernel based methods [26], pattern classification methods [27], Convolution Neural Networks (CNN) [28], fuzzy approaches [29], Analysis of Variance (ANOVA), and *K*-Nearest Neighbour (KNN) [30] were proposed in the literature. Using ant colony optimization, a hybrid gene selection approach was proposed by Sharbaf et al. [31]. For the cancer classification data on gene expression data, PSO and DT classifiers were implemented by Chen et al. [32]. For gene selections, the various techniques reported in literature are utilizing multiobjective algorithms [33], a hybrid binary Imperialist Competition Algorithm (ICA), and tabu search approach [34], a binary differential evolution algorithm [35], a simplified swarm optimization using a Social Spider Optimization (SSO) algorithm [36], Artificial Bee Colony (ABC) [37], Binary PSO [38], novel rule-based algorithm [39], and Shuffled Leap Frog Algorithm (SLFA) [40], and it has been well explored. However, in this paper, other suitable swarm intelligence techniques have been explored and analyzed comprehensively. The organization of the paper is as follows.  In Section 2, the materials and methods followed by the gene selection techniques are explained.  In Section 3, the optimization techniques for gene selection are explained, and in Section 4, the classification techniques are explained followed by the results and discussion in Section 5 and conclusion in Section 6.

## 2. Materials and Methods

For the lung cancer classification, a lung Harvard 2 dataset was utilized, which is publicly available online [41]. The dataset has 181 samples with 150 Adenocarcinoma (ADCA) and 31 Malignant Pleural Mesothelioma (MPM). The dataset is tabulated in Table 1.

The pictorial representation of the work is shown in Figure 1.

### 2.1. Gene Selection Techniques

The gene selection techniques utilized in this paper are Information Gain, Relief-F, Chi-square statistic, and T-statistic. The discretization of the attribute values is done before using chi-square, information gain, and other feature selection methods. The main intention of utilizing the gene selection techniques is to select the most important genes from 12,533 genes. Here, in our work, we have selected 1000 important genes after the gene selection process through the following techniques.

#### 2.1.1. Information Gain

It is used generally as an attribute selection criteria while dealing with decision trees; hence, it is used as a gene selection technique too [7]. Assume the class set *S*={*S*_*x*_}, where *x*=1,2,…, *l*. For every feature *Y*_*j*_, the Information Gain is expressed as

(1) $$\begin{array}{c} \text{InfoGain}\left(Y_{j}\right)=H\left(S\right)-H\left(\frac{S}{Y_{j}}\right), \end{array}$$

where *H*(*S*)=−∑_*s*∈*S*_*p*(*s*)log_2_  *p*(*s*) and

(2) $$\begin{array}{c} H\left(\frac{S}{Y_{j}}\right)=-\sum_{y\in Y_{j}}p\left(y\right)\sum_{s\in S}p\left(\frac{s}{y}\right)\log_{2}\;p\left(\frac{s}{y}\right). \end{array}$$

Only for discrete features, Information Gain is used widely, and therefore prior to computing Information Gain, the discretization of numeric features should be done. Depending on the large values of information gain, the selection of features are done.

#### 2.1.2. Relief–F

For dealing with multiclass, noisy, and incomplete datasets, Relief-F is introduced, and it is an extension of Relief algorithm [7]. To each feature, a relevance weight is assigned. The selection of a random sample instance *I* is done from *n* sample instances. Based on the basic differences between the selected instance *I* and its neighboring instance represented as *Q* and termed as hit and different class termed as nearest miss represented by *N*(*S*), the updating of the relevance features is done. The features that discriminate the instance from various neighbors of the surrounding classes are given more weight. By analyzing the average contribution of neighboring nearest misses *N*(*S*), the updating of the weights is done. The prior probability of each class is considered by the average contribution. The updating of the weight of *j*^th^ feature *Y*_*j*_ is as follows:

(3) $$\begin{array}{c} w_{j}=w_{j}-\frac{\Psi \left(Y_{j},I,Q\right)}{n}+\sum_{S=S_{I}}\frac{P\left(S\right)*\Psi \left(Y_{j,}I,N\left(s\right)\right)}{n}, \end{array}$$

where the distance between sample instances (*I*) and the nearest hit (*Q*) or nearest miss *N*(*S*) is calculated by the function Ψ(*Y*_*j*,_*I*, *Q*).

#### 2.1.3. Chi-Square Statistic

With respect to the classes, for each feature, the value of *χ*^2^ statistic is computed [7]. Before computing *χ*^2^ statistic, the discretization of the numeric attributes is done. For every feature, *Y*_*j*_, *χ*^2^ statistic is computed as

(4) $$\begin{array}{c} \chi^{2}=\sum_{y\in Y_{j}}\sum_{s\in S}\frac{{\left(n_{\left(y\in Y_{j}\&s\in S\right)}-e_{\left(y\in Y_{j}\&s\in S\right)}\right)}^{2}}{e_{\left(y\in Y_{j}\&s\in S\right)}}, \end{array}$$

where *n*_(*y* ∈ *Y*_*j*_&*s* ∈ *S*)_ represent the number of samples in *Y*_*j*_ for class *s* whose value is *y*. The definition of expected frequency is expressed as

(5) $$\begin{array}{c} e_{\left(y\in Y_{j}\&s\in S\right)}=\frac{n_{y\in Y_{j}}\times n_{s\in S}}{n}, \end{array}$$

where the number of samples in *Y*_*j*_ with value *y* is denoted by *n*_*y*∈*Y*_*j*__; *n*_*s*∈*S*_ indicates the number of samples of class *s*. The total number of samples is expressed by *n*. Based on the sorted value of *χ*^2^ statistic, the selection of features is done.

#### 2.1.4. *T*-Statistic

This is a famous gene selection technique and quite popular in two-class problems [7]. Every sample can be classified into either class *S*_1_ or class *S*_2_. For every feature *Y*_*j*_, the computation of t-statistic is expressed as

(6) $$\begin{array}{c} t\left(Y_{j}\right)=\frac{\left|\mu_{j1}-\mu_{2}\right|}{\sqrt{\left(\sigma_{j1}^{2}/n_{1}\right)+\left(\sigma_{j2}^{2}/n_{2}\right)}}, \end{array}$$

where *μ*_*jk*_ indicates the mean of the *j*^th^ feature for class *S*_*k*_. The “*k*” indicates the class index, i.e., *k*=1 or *k*=2.

Once the t-statistic value for each feature is computed, then it is sorted out in a descending order, so that the important features can be selected.

## 3. Optimization Techniques

The shortlisted 1000 genes will undergo again a secondary feature selection methodology to select the best 50 genes, 100 genes, and 200 genes by means of utilization of optimization techniques. The second level feature selection is done using the five optimization algorithms as follows.

### 3.1. Grasshopper Optimization Algorithm

In many engineering optimization problems, this algorithm is widely used. Based on the biggest swarms of all creatures, one of the recently proposed naturally inspired algorithms is GO [42]. Severe damage to the crops is caused by the herbivores grasshopper. The grasshopper has a swarming behavior, and it depends on both adults and nymphs. Soft plants and succulents are fed by the nymph, which rolls on the ground continuously. In search of food, the adult grasshopper can jump to a very high extent, and so, it will have a very large area to explore. The observation of both types of movement such as slow movement and abrupt movement has been achieved, which indicates that exploitation and exploration are possible. For the grasshopper, the swarming behavior is represented mathematically as

(7) $$\begin{array}{c} Q_{j}=A_{j}+F_{j}+B_{j}, \end{array}$$

where *Q*_*j*_ represents the position of the *j*^th^ grasshopper, *A*_*j*_ represents the social interaction, *F*_*j*_ represents the gravity force in the *j*^th^ grasshopper, and *B*_*j*_ represents the wind advection. The representation of social interaction *A*_*j*_ is given as

(8) $$\begin{array}{c} A_{j}=\sum_{k=1,k\neq j}^{N}a\left(d_{jk}\right){\hat{d}}_{jk}, \end{array}$$

where *d*_*jk*_=|*q*_*k*_ − *q*_*j*_| represents the distance between the *j*^th^ and *k*^th^ grasshopper and ${\hat{d}}_{jk}=\left(q_{k}-q_{j}\right)/\left(d_{jk}\right)$ represents a unit vector from the *j*^th^ grasshopper to the *k*^th^ grasshopper. The social forces are expressed by the function “*a*” and are expressed as

(9) $$\begin{array}{c} a\left(s\right)=ge^{\left(-\left(s/l\right)\right)}-e^{-s}, \end{array}$$

where the intensity of the attraction is represented as *g* and the attractive length scale is expressed by *l*. In terms of social interaction, three types of regions are created by the grasshoppers in search of food, that is, attraction zone, comfort zone, and repulsion region. Strong forces cannot be applied by the function “*a*” when the distance is large between grasshoppers. To resolve this, the *F* component in (7) is expressed as

(10) $$\begin{array}{c} F_{j}=-f{\hat{e}}_{f}, \end{array}$$

where the *f* represents the gravitational constant and ${\hat{e}}_{f}$ indicates a unity vector progressing towards the Earth center. The computation of *B* component is as follows:

(11) $$\begin{array}{c} B_{j}=v{\hat{e}}_{u}, \end{array}$$

where *v* represents the constant drift and ${\hat{e}}_{u}$ represents a unity vector in the wind direction. If the values of *a*, *F* and *B* are substituted in (7), then

(12) $$\begin{array}{c} Q_{j}=\sum_{K=1,K\neq j}^{N}a\left(\left|q_{k}-q_{j}\right|\right)\frac{q_{k}-q_{j}}{d_{jk}}-f{\hat{e}}_{f}+v{\hat{e}}_{u}, \end{array}$$

where *a*(*s*) is given by (9) and the number of grasshoppers is represented by *N*. To solve optimization problems, a revised version of this formula is used as

(13) $$\begin{array}{c} Q_{j}^{d}=c\left(\sum_{k=1k\neq j}^{N}c\frac{v_{bd}-l_{bd}}{2}a\left(\left|q_{k}^{d}-q_{j}^{d}\right|\right)\frac{q_{k}-q_{j}}{d_{jk}}\right)+{\hat{T}}_{d}, \end{array}$$

where *v*_*bd*_ represents the upper bound and *l*_*bd*_ represents the lower bound in the *D*^th^ dimension. In the target, the value of the *D*^th^ dimension is represented by ${\hat{T}}_{d}$. To shrink the three worms, the decreasing coefficient is “*c*.” Only towards a target the wind direction is progressed always. While the food is a searched form, adults start jumping in the air, and nymphs move on rolling in the ground creating both cases of exploration and exploitation. By reducing the parameter *c* in the below equation, one can balance both these two in proportion to the total number of iterations. Its computation is done as

(14) $$\begin{array}{c} c=c_{\max}-i\left[\frac{c_{\max}-c_{\min}}{I}\right], \end{array}$$

where the maximum value is represented as *c*_max_, minimum value is represented as *c*_min_, *i* denotes the current iteration, and *I* represents the maximum number of iterations.

### 3.2. Moth Flame Optimization Algorithm

Based on the simulation of moth behavior for this special movement method during nighttime, Moth flame optimization algorithm was developed [43]. For the purpose of navigation or movement, a mechanism termed as transverse orientation is utilized. By maintaining a standard angle with reference to the moon, moth flies, which is a very effective methodology for travelling by distances in a straight path, as the distance between the moon and the moth is very far away. This kind of methodology is adopted, so that moth flies along a very straight path at nighttime. It is a general observation that the moths fly around the lights in a spiral manner. The artificial lights can easily trick the moths to exhibit such behavior. As the light lies with close proximity to the moon, a spiral fly of moths is caused due to the maintenance of a similar angle to the light source. In this algorithm, the representation of the set of moths is done as a matrix *A*. For the storage of all the corresponding fitness values, there is an array OA for all the moths. In this algorithm, the second key component is the flames. Now, again, a matrix *B* similar to the moth matrix is considered. For the storage of all the corresponding fitness values, there is an array OB for all the flames. The global optimal of the optimization problem is approximated by the MFO algorithm by a three-tuple process as follows:

(15) $$\begin{array}{c} \text{MFO}=\left(C,D,K\right). \end{array}$$

A random population of moths with its corresponding fitness value is denoted by a function *C*. In this function, the methodical model is expressed as

(16) $$\begin{array}{c} C:\phi ⟶\left\{A,OA\right\}. \end{array}$$

The movement of the moths around the search space is determined by the function *D* which is the primary function. The matrix of *A* is received by this function and eventually returns the updated one as

(17) $$\begin{array}{c} D:A⟶A. \end{array}$$

The *K* function remains true if termination criterion is satisfied and false if the termination criterion is not satisfied.

(18) $$\begin{array}{c} K:A⟶\left\{\text{true,false}\right\}, \end{array}$$

With *C*, *D*, and *K*, the general framework of the MFO is expressed as follows:

 
*A*=*C*()( );
  while *K*(*A*) is equal to false
 
*A*=*D*(*A*);
  end

Until the *K* function returns true, the *D* function is run iteratively after the initialization. To simulate the moth behavior mathematically, the updating of the position of every moth is updated with respect to a flame using the following equation:

(19) $$\begin{array}{c} A_{c}=F\left(A_{c},B_{g}\right), \end{array}$$

where *A*_*c*_ indicates the *c*^th^ moth, *B*_*g*_ specifies the *g*^th^ flame, and *F* represents the spiral function.

Subject to the following conditions, the utilization of any type of spiral can be done using the three conditions as follows:

1. The initial point of the spiral should begin from the moth
2. The final point of the spiral should be the flame position
3. The range of spiral fluctuation should not exceed the search space

For the MFO algorithm, the logarithmic spiral is defined as

(20) $$\begin{array}{c} F\left(A_{c},B_{g}\right)=J_{c}\cdot e^{hk}\cdot \;\cos\left(2\pi k\right)+B_{g}, \end{array}$$

where *J*_*c*_ specifies the distance of the *c*^th^ moth for the *g*^th^ flame, *h* denotes a constant for defining the shape of a logarithmic spiral, and *k* is a random number in [−1, 1].

The computation of *J* is done as follows:

(21) $$\begin{array}{c} J_{c}=\left|B_{g}-A_{c}\right|, \end{array}$$

where *A*_*c*_ indicates the *c*^th^ moth, *B*_*g*_ specifies the *g*^th^ flame, and *J*_*c*_ specifies the distance of the *c*^th^ moth for the *g*^th^ flame.

The spiral flying path of the moth is expressed by (20). From this equation, with respect to a flame, the next position of a moth is explained. In the spiral equation, the *k* parameters defer the next position of the moth with reference to its proximity or closeness to the flame. While the position is updated, it only regains a moth to progress towards a flame; thereby, it may be trapped in local optima fastly. Each moth is obliged to update its position using only one of the flames to prevent such situations. The position updating of moths with respect to “*n*” various locations in the search space may sometimes denote the exploitation of most promising solutions.

(22) $$\begin{array}{c} \text{flame number}=\text{round}\left[N-I*\frac{N-1}{K}\right], \end{array}$$

where *I* denotes the current number of iterations, *N* denotes the maximum number of flames, and *K* specifies the maximum number of iterations. To balance the exploration and exploitation of the search space, there is a gradual decrease in the number of flames. The general steps of the *D* function are described in Algorithm 1.

As projected in the algorithm, unless the *K* function returns true, the *D* function is executed. Once the *D* function is terminated, the best moth returns, as it is shown as the best attained optimum approximation value.

### 3.3. Bacterial Foraging Optimization Algorithm

The three main mechanisms are present in the classical BFO, that is, chemotaxis process, reproduction process, and elimination-dispersal process [44].

#### 3.3.1. Chemotaxis Process

Here, a tumble indicates a unit walk with random direction, and a run indicates a unit walk with the similar direction in the last step. Assuming *θ*^*a*^(*b*, *c*, *d*) indicates the bacterium at *b*^th^ chemotactic, *c*^th^ reproductive, and *d*^th^ elimination-dispersal method. *R*(*a*) is considered as the run-length unit parameter is the chemotactic step size during every tumble or run. The movement of the *a*^th^ bacterium in every computational chemotactic step is expressed as

(23) $$\begin{array}{c} \theta^{a}\left(b+1,c,d\right)=\theta^{a}\left(b,c,d\right)+R\left(a\right)\frac{\Delta \left(a\right)}{\sqrt{\Delta^{T}\left(a\right)\Delta \left(a\right)}}, \end{array}$$

where Δ(*a*) represents the direction vector of the *b*^th^ chemotactic step. Δ(*a*) is the same as the final chemotactic step if the bacterial movement is run; or else Δ(*a*) becomes a random vector, where specific elements lie in the range of [−1, 1]. A step fitness indicated as *B*(*a*, *b*, *c*, *d*) is evaluated with the activity of both run or tumble assumed and considered at each step during the chemotaxis process.

#### 3.3.2. Reproduction Process

During its lifetime, the sum of the step fitness is calculated as the health status of each bacterium as ∑_*b*=1_^*N*_*r*_^*B*(*a*, *b*, *c*, *d*), where *N*_*r*_ represents the maximum step in a chemotaxis process. Based on the health status, the sorting of the bacteria is done in a reverse order. Only the first half of population lives/survives in the reproductive step. The living bacterium divides into two identical ones, and they are kept in the same places, and so the population of bacteria keeps constant.

#### 3.3.3. Elimination and Dispersal Process

A basis for local search is provided by the chemotaxis, and the convergence is sped up by the reproduction process. Using the classical BFO, this situation has been simulated to a large extent. For searching of global optima, only chemotaxis and reproduction are not enough. Around the local optima, the bacteria may get stuck and to eliminate the accidents of being trapped into local optima easily and gradually, the diversity of the BFO changes. Only after a certain number of reproductive processes, the dispersion event happens. Then, based on a probability *P*_*pr*_, some bacteria are chosen to be killed and shifted to another position within a particular environment. The step by step procedure is explained in Algorithm 2.

### 3.4. Krill Herd Optimization Algorithm

Based on the simulation of the herding of krill swarms, a famous metaheuristic algorithm for solving optimal problems is KH optimization algorithm [45]. The herding of the skill swarms is usually in response to a certain environmental and biological process. In a 2D space, the time-dependent position of an individual krill is decided by 3 primary actions, that is,

- Movement which influences or influenced by other krill individuals.
- Foraging actions
- Random diffusion

In a d-dimensional decision space, the following Lagrangian model is adopted by the KH algorithm as

(24) $$\begin{array}{c} \frac{\text{d}Z_{j}}{\text{d}t}=M_{j}+G_{j}+D_{j}, \end{array}$$

where *M*_*j*_ is the motion led by other krill individuals, *G*_*j*_ is the foraging motion, and *D*_*j*_ is the physical diffusion of the *j*^th^ krill individual.

The krill individuals affecting the other movement are represented by the direction of motion *α*_*j*_ and it is computed by the target swarm density, a local swarm density, and a repulsive swarm density. The movement for a krill individual is defined as follows:

(25) $$\begin{array}{c} M_{j}^{\text{new}}=M^{\max}\alpha_{j}+v_{m}M_{j}^{\text{old}}. \end{array}$$

The maximum induced speed is represented by *M*^max^, the inertia weight of the motion induced in [0, 1] is represented as *v*_*m*_ and the latest motion induced is represented by *M*_*j*_^old^.

With the help of two main components, the estimation of foraging motion is done. The first one is the food location, and the second one is the basic knowledge about the food location. The motion is approximately formulated for the *j*^th^ krill individual as follows:

(26) $$\begin{array}{c} G_{j}=W_{g}\beta_{j}+v_{g}G_{j}^{\text{old}}, \end{array}$$

where

(27) $$\begin{array}{c} \beta_{j}=\beta_{j}^{\text{food}}+\beta_{j}^{\text{best}}, \end{array}$$

where the foraging speed is represented by *W*_*g*_. The inertia weight of the foraging motion between 0 and 1 is represented as *v*_*g*_ and *G*_*j*_^old^ is the last foraging action.

A random process is modelled to the random diffusion of the krill individuals. In terms of both a random directional vector and maximum diffusion speed, the description of the motion can be done. It is represented as follows:

(28) $$\begin{array}{c} D_{j}=D^{\max}\delta , \end{array}$$

where the maximum diffusion speed is *D*^max^, the random directional vector is *δ* and its arrays are random values in the range of [−1, 1]. Utilizing various motion parameters during the time and based on the above-mentioned movements, using the following equation, the position vector of a krill individual from the time interval *t* to *t*+Δ*t* is given as

(29) $$\begin{array}{c} Z_{j}\left(t+\Delta t\right)=Z_{j}\left(t\right)+\Delta t\frac{\text{d}Z_{j}}{\text{d}t}, \end{array}$$

Δ*t* is regarded as the most important term and based on the specific type of optimization, the parameters can be fine-tuned. The scalar factor of the speed vector is assumed because of Δ*t* parameter.

### 3.5. Artificial Fish Swarm Optimization Algorithm

It is a famous Swarm Intelligence technique, which is helping to solve the optimization problem by utilizing the behavior of artificial fishes like imitating swarming process, chasing process, and preying behaviors [46]. Assume *A*_*p*_ is the current position of one artificial fish and *A*_*w*_ is the viewpoint of artificial fish at one specific moment. The visual scope of every individual is expressed as *Vis*; therefore, within *Vis* of *A*_*p*_ be the fishes *A*_*y*_ and *A*_*z*_. The largest step of artificial fish is assumed as step and the congestion factor of the fish swarm is expressed as *δ*. The food concentration factor is highly proportional to the fitness function *f*(*A*). In the fish swarm, the behavior patterns are expressed as follows:

#### 3.5.1. Swarming Behavior

If *f*(*A*_*s*_) > *f*(*A*_*p*_), then *A*_*s*_ is the central point inside the *Vis* of the point *A*_*p*_ and so the execution of swarming behavior is done easily. Assume *A*_*s*_ as *A*_*w*_ and so, the fish at *A*_*p*_ will progress towards the point *A*_*s*_.

#### 3.5.2. Chasing Behavior

The point (expressed by *A*_max_), which has the best objective function value, is present inside the visual satisfying the criterion *f*(*A*_max_) > *f*(*A*_*p*_) and if there is less crowd in the visual of *A*_*p*_ , then the execution of chasing behavior is done. Consider *A*_max_ as *A*_*w*_ and so, the fish at *A*_*p*_will progress towards the point *A*_max_.

#### 3.5.3. Preying Behavior

Under the following situations, preying behavior is tried.

- *f*(*A*_*q*_) > *f*(*A*_*p*_), *f*(*A*_max_) < *f*(*A*_*p*_) and there is less or no crowd in the *Vis*
- Alternatively, if the visual is crowded, then the random selection of a point *A*_*q*_ inside the visual of *A*_*p*_ is done.

The preying behavior is executed if *f*(*A*_*q*_) > *f*(*A*_*p*_). Assume *A*_*q*_ as *A*_*w*_ and so, the fish at *A*_*p*_ will progress towards the point *A*_*q*_. Otherwise, with its visual limit, it will move a step in a random fashion.

In each iteration, the best solution obtained is termed as “board.” The search process can be terminated after the specified iterations, and the result present on the board is considered as the final solution. The position updating for the artificial preying fishes is formulated as

(30) $$\begin{array}{c} A_{\text{next}}=A_{p}+\text{rand}\cdot \frac{\text{step}\times \left(A_{q}-A_{p}\right)}{\text{norm}\left(A_{q}-A_{p}\right)}, \end{array}$$

where the next position of artificial fish is termed as *A*_next_. The current position of the artificial fish is expressed as *A*_*p*_ and the position having a better objective function value is *A*_*q*_. The random number is expressed as rand and it is in the range of [−1, 1]. Between the two position vectors, the distance is expressed as norm(*A*_*q*_ − *A*_*p*_). The position updating for the artificial swarm fishes can be done as

(31) $$\begin{array}{c} A_{\text{next}}=A_{p}+\text{rand}\cdot \frac{\text{step}\times \left(A_{s}-A_{p}\right)}{\text{norm}\left(A_{s}-A_{p}\right)}. \end{array}$$

The position updating for the artificial chasing fishes is formulated as

(32) $$\begin{array}{c} A_{\text{next}}=A_{p}+\text{rand}\cdot \frac{\text{step}\times \left(A_{\max}-A_{p}\right)}{\text{norm}\left(A_{\max}-A_{p}\right)}. \end{array}$$

## 4. Classification Procedures

The optimized values or the best gene values obtained after the second level optimization techniques are classified using NBC, Decision trees, SVM, and KNN algorithms. The Performance Analysis of Classifiers in terms of Classification accuracies with GO, MHO, BFO, KHO, and AFSO for different gene selection techniques using 50–200 selected genes is done here.

### 4.1. Naïve Bayesian Classifier

It is a famous probabilistic algorithm, where, given the class, the feature values based on Bayes rule are conditionally independent [47]. If a new sample observation is given, the assignment of the classifier to the class having the maximum conditional probability estimate is done.

### 4.2. Decision Tree

A famous rule-based classifier is DT, where leaf nodes represent classification outcomes and non-leaf nodes represent selected attributes [48]. A classification rule is reflected by the path from the root to a leaf node. The J4.8 algorithm is used here.

### 4.3. Support Vector Machine

The SVM analyzes the input data as two unique sets of vector in a p-dimensional space initially [49]. Then, in that space, a separate hyperplane is constructed, so that the margin is maximized between the two data sets. The SVM is utilized with SVM Polynomial kernels for training purposes.

### 4.4. KNN Algorithm

One of the famous instance-based classifiers is KNN [50]. The class label of a new testing sample is decided by the classifier. It is done by considering the majority of classes of its K closest neighbors dependent on their Euclidean distance. Here, the value of *K* is assigned to be 4.

## 5. Results and Discussion

It is classified with a 10-fold cross-validation method, and its performance is shown in the tables. The mathematical formulae for computing the Performance Index (PI), Sensitivity, Specificity, and Accuracy are mentioned in literature and using the same, the values are computed and exhibited. PC is Perfect Classification; MC is Missed Classification; and FA is False Alarm in the following expressions.

The sensitivity is expressed as

(33) $$\begin{array}{c} \text{Sensitivity}=\frac{\text{PC}}{\text{PC}+\text{FA}}\times 100. \end{array}$$

Specificity is expressed as

(34) $$\begin{array}{c} \text{Specificity}=\frac{\text{PC}}{\text{PC}+\text{MC}}\times 100. \end{array}$$

Accuracy is expressed as

(35) $$\begin{array}{c} \text{Accuracy}=\frac{\text{Sensitivity}+\text{Specificity}}{2}. \end{array}$$

Performance Index (PI) is expressed as

(36) $$\begin{array}{c} \text{PI}=\left(\frac{\text{PC}-\text{MC}-\text{FA}}{\text{PC}}\right)\times 100. \end{array}$$

Table 2 shows the performance analysis of classifiers for classification accuracy parameter with GO method for different gene selection techniques. As indicated in Table 2 that SVM classifier with 100 selected genes in Relief F test method and NBC with information gain method for 100 genes attained higher accuracy of 98.96%. The lower accuracy of 76% is thrown out by KNN classifier in all three statistical methods.

Table 3 indicates the performance analysis of classifiers for classification accuracy with MFO method for different gene selection techniques. As shown in Table 3, DT classifier with 50 selected genes in Relief F test method reached higher accuracy of 98.012%. The lower accuracy of 78.125% is depicted by SVM classifier with 100 genes selected in relief F test method. The lower accuracy of SVM is due to the presence of outlier in the gene samples.

Table 4 demonstrates the performance analysis of classifiers for classification accuracy with BFO method for different gene selection techniques. From Table 4, it is identified that DT classifier with 50 selected genes in Chi-square test method reached higher accuracy of 98.56%. The lower accuracy of 82.24% is shown by SVM classifier with 100 genes selected in information gain method. Across the gene samples, all the classifiers performed well in this BFO method.

Table 5 reveals the performance analysis of classifiers for classification accuracy with KHO method for different gene selection techniques. Table 5 shows that SVM classifier with 50 selected genes in Relief F test method reached higher accuracy of 98.38%, as the number of selected genes increased gradually and given to SVM classifiers, which reported lower accuracy of 77.47% with 200 genes selected in Relief F test method.

Table 6 reports the performance analysis of classifiers for classification accuracy with AFSO method for different gene selection techniques. As indicated in Table 6, DT classifier with 100 selected genes in Relief F test method reached the highest accuracy of 99.10%. The NBC classifier is settled at the lower accuracy of 77.08% with 200 selected genes for Relief F test method.

Table 7 signifies the performance analysis of classifiers for classification PI parameter with GO method for different gene selection techniques. As shown in Table 7, SVM classifier with 100 selected genes in Relief F test method and NBC with information gain for 100 genes attained higher PI of 97.87%. The lower PI of 7.69% is indicated by KNN classifier in all three statistical methods.

Table 8 demonstrates the performance analysis of classifiers for classification PI with MFO method for different gene selection techniques. As shown in Table 8, DT classifier with 50 selected genes in Relief F test method reached higher PI of 95.85%. The lower PI of 22.22% is indicated by SVM classifier with 100 genes selected in Relief F test method. The lower PI of SVM is due to the presence of outlier genes in the samples.

Table 9 represents the performance analysis of classifiers PI with BFO method for different gene selection techniques. From Table 9, it is known that DT classifier with 50 selected genes in Chi-square test method reached higher PI of 97.009%. The lower PI of 45.09% is indicated by SVM classifier with 100 genes selected in information gain method. Across the gene samples, all the classifiers performed well in this BFO.

Table 10 exposes the performance analysis of classifiers for classification PI with KHO method for different gene selection techniques. Table 10 reported that SVM classifier with 50 selected genes in Relief F test method reached higher PI of 96.68%, as the number of selected genes increased gradually and given to SVM classifiers, which reported lower PI of 17.93% with 200 genes selected in Relief-F test method.

Table 11 details the performance analysis of classifiers for classification PI with AFSO method for different gene selection techniques. As indicated in Table 11, DT classifier with 100 selected genes in Relief F test method reached the highest PI of 98.16%. The NBC classifier depicts lower PI of 15.36% with 200 selected genes for the same Relief F test method.

## 6. Conclusion and Future Work

One of the most prominent lethal factors for human beings nowadays is cancer. The best chances of suitable treatment can sometimes be missed due to mistaken diagnosis. The accuracy of cancer diagnosis with machine learning along with clinical tests is very helpful in the treatment of cancer. Microarray expression data is highly redundant and with respect to most number of classes, the genes present are uninformative. Therefore, it is a critical necessity to select the best feature genes for the analysis of cancer. Out of a large dataset, the techniques should be capable of identifying a subset of most informative genes in a robust manner. In this work, a comprehensive analysis of lung cancer classification with the help of feature selection and optimization techniques is done. The best results are obtained when Relief-F test is computed with AFSO and classified with Decision Trees classifier for hundred genes, and a highest classification accuracy of 99.10% is obtained. Future works aim to work with other feature selection techniques and a variety of optimization techniques classified with deep learning techniques for effective classification of lung cancer.

## Figures and Tables

**Figure 1:** Pictorial representation of the work.

**Algorithm 1:** D function execution and termination.

**Algorithm 2:** BFO.

**Table 1:** Dataset details.

Dataset	Number of genes	Class 1 (ADCA)	Class 2 (MPM)	Total samples
Lung Harvard 2	12533	150	31	181

**Table 2:** Performance analysis of classifiers in terms of classification accuracies (%) with Grasshopper optimization for different gene selection techniques using 50–200 selected genes.

Method	NBC			DT			SVM			KNN		
Genes selected	50	100	200	50	100	200	50	100	200	50	100	200
Information gain	82.29	98.96	76	78.12	83.59	83.59	76	83.59	77.08	76	76	77.08
Relief–F test	85.93	91.67	83.59	83.59	78.12	89.6	78.12	98.96	95.83	87.5	78.12	77.08
Chi-square test	97.91	77.08	83.59	95.83	93.75	77.08	82.29	83.59	91.67	76	77.08	83.59
*T* statistic test	77.08	82.29	82.29	97.91	95.83	78.12	83.59	93.75	95.83	77.08	76	85.93

**Table 3:** Performance analysis of classifiers in terms of classification accuracies (%) with Moth flame optimization for different gene selection techniques using 50–200 selected genes.

Method	NBC			DT			SVM			KNN		
Genes selected	50	100	200	50	100	200	50	100	200	50	100	200
Information gain	96.34	89.6	93.75	85.93	83.59	93.26	91.67	97.91	89.6	89.6	83.59	95.83
Relief–F test	93.75	82.29	91.67	98.01	97.91	86.19	85.93	78.12	95.83	82.29	97.91	89.6
Chi-square test	93.75	93.75	90.74	91.67	85.93	84.10	97.91	86.40	85.93	85.93	97.91	91.67
*T* statistic test	85.93	91.67	95.83	85.93	93.75	84.75	96.15	85.93	91.67	85.93	85.93	97.91

**Table 4:** Performance analysis of classifiers in terms of classification accuracies (%) with Bacterial foraging optimization for different gene selection techniques using 50–200 selected genes.

Method	NBC			DT			SVM			KNN		
Genes selected	50	100	200	50	100	200	50	100	200	50	100	200
Information gain	97.91	96.85	91.64	95.83	85.93	85.93	85.02	82.24	89.92	85.93	87.12	93.75
Relief–F test	97.91	93.75	89.6	89.6	91.67	83.59	97.91	83.81	87.30	95.83	97.91	97.91
Chi-square test	93.75	89.6	91.67	98.56	90.53	97.33	97.72	85.93	97.91	97.91	95.83	95.83
*T* statistic test	91.67	93.75	85.93	84.41	95.83	98.04	86.71	97.91	84.95	95.83	93.75	89.6

**Table 5:** Performance analysis of classifiers in terms of classification accuracies (%) with Krill Herd optimization for different gene selection techniques using 50–200 selected genes.

Method	NBC			DT			SVM			KNN		
Genes selected	50	100	200	50	100	200	50	100	200	50	100	200
Information gain	97.91	91.67	81.57	86.58	89.6	96.76	91.89	93.75	97.91	92.05	91.40	96.92
Relief–F test	89.6	97.91	83.59	82.29	85.93	87.37	98.38	79.21	77.47	83.46	90.97	84.25
Chi-square test	93.75	93.27	81.72	97.12	82.59	92.12	88.55	78.99	98.69	87.88	78.61	88.91
*T* statistic test	95.83	97.91	91.67	95.83	96.93	95.83	94.72	85.06	96.67	86.73	88.03	98.96

**Table 6:** Performance analysis of classifiers in terms of classification accuracies (%) with Artificial fish swarm optimization for different gene selection techniques using 50–200 selected genes.

Method	NBC			DT			SVM			KNN		
Genes selected	50	100	200	50	100	200	50	100	200	50	100	200
Information gain	90.24	91.67	89.05	88.41	86.82	81.03	94.90	93.75	93.75	93.75	89.6	93.75
Relief–F test	95.96	85.93	77.08	89.79	99.10	86.42	95.83	97.91	97.91	89.6	78.59	80.56
Chi-square test	82.59	83.48	78.12	84.10	95.34	94.61	95.83	98.63	93.75	94.49	97.91	84.39
*T* statistic test	93.75	89.75	87.5	86.78	92.29	89.33	89.6	97.91	97.91	95.83	94.79	97.91

**Table 7:** Performance analysis of classifiers in terms of PI (%) with Grasshopper optimization for different gene selection techniques using 50–200 selected genes.

Method	NBC			DT			SVM			KNN		
Genes selected	50	100	200	50	100	200	50	100	200	50	100	200
Information gain	45.16	97.87	7.69	22.22	51.16	51.16	7.69	51.16	15.36	7.69	7.69	15.36
Relief–F test	60.87	80.01	51.163	51.163	22.22	78.93	22.22	97.87	91.58	66.66	22.22	15.36
Chi-square test	95.65	15.36	51.163	91.58	85.7	15.36	45.16	51.16	80.01	7.69	15.36	51.16
*T* statistic test	15.36	45.16	45.16	95.65	91.58	22.22	51.16	85.7	91.58	15.36	7.69	60.87

**Table 8:** Performance analysis of classifiers in terms of PI (%) with Moth flame optimization for different gene selection techniques using 50–200 selected genes.

Method	NBC			DT			SVM			KNN		
Genes selected	50	100	200	50	100	200	50	100	200	50	100	200
Information gain	92.45	78.93	85.7	60.87	51.16	84.31	80.01	95.65	78.93	78.93	51.16	91.58
Relief-F test	85.7	45.16	80.01	95.85	95.65	61.14	60.87	22.22	91.58	45.16	95.65	78.93
Chi-square test	85.7	85.7	77.62	80.01	60.87	53.35	95.65	62.50	60.87	60.87	95.65	80.01
*T* statistic test	60.87	80.01	91.58	60.87	85.7	56.08	92.17	60.87	80.01	60.87	60.87	95.65

**Table 9:** Performance analysis of classifiers in terms of PI (%) with Bacterial foraging optimization for different gene selection techniques using 50–200 selected genes.

Method	NBC			DT			SVM			KNN		
Genes selected	50	100	200	50	100	200	50	100	200	50	100	200
Information gain	95.65	93.17	79.93	91.58	60.87	60.87	57.22	45.09	78.31	60.87	64.03	85.7
Relief-F test	95.65	85.7	78.93	78.93	80.01	51.16	95.65	52.11	63.85	91.58	95.65	95.65
Chi-square test	85.7	78.93	80.01	97.00	77.11	94.45	94.96	60.87	95.65	95.65	91.58	91.58
*T* statistic test	80.01	85.7	60.87	52.98	91.58	95.92	63.76	95.65	56.00	91.58	85.7	78.93

**Table 10:** Performance analysis of classifiers in terms of PI (%) with Krill Herd optimization for different gene selection techniques using 50–200 selected genes.

Method	NBC			DT			SVM			KNN		
Genes selected	50	100	200	50	100	200	50	100	200	50	100	200
Information gain	95.65	80.01	39.87	62.47	78.93	93.44	80.36	85.7	95.65	81.07	79.21	93.28
Relief-F test	78.93	95.65	51.16	45.16	60.87	64.68	96.68	28.94	17.93	50.06	78.04	53.72
Chi-square test	85.7	84.41	42.31	93.60	46.56	81.00	72.79	27.54	97.28	68.96	24.01	74.91
*T* statistic test	91.58	95.65	80.01	91.58	93.22	91.58	88.45	57.42	92.69	63.08	62.83	97.87

**Table 11:** Performance analysis of classifiers in terms of PI (%) with Artificial fish swarm optimization for different gene selection techniques using 50–200 selected genes.

Method	NBC			DT			SVM			KNN		
Genes selected	50	100	200	50	100	200	50	100	200	50	100	200
Information gain	77.67	80.01	75.76	72.02	64.12	37.59	88.01	85.7	85.7	85.7	78.93	85.7
Relief-F test	91.26	60.87	15.36	78.55	98.16	62.67	91.58	95.65	95.65	78.93	25.11	35.42
Chi-square test	46.56	50.67	22.22	53.37	90.08	88.09	91.58	97.14	85.7	87.6	95.65	54.61
*T* statistic test	85.7	78.67	66.66	65.91	82.65	77.2	78.93	95.65	95.65	91.58	88.64	95.65

## Data Availability

The data along with the program codes will be available to genuine researchers upon request to the corresponding author.
